The article "Ischemic Stroke With Hemorrhagic Conversion in a Case of Lyme Neuroborreliosis" was published in 2022. Journal: Cureus.

# Ischemic Stroke With Hemorrhagic Conversion in a Case of Lyme Neuroborreliosis

**DOI:** 10.7759/cureus.28028

**Published:** 2022-08-15

**Authors:** Srinandan Sathi, Daniel Kim, Patrick Duplan, Paul Kim, Carl Shenkamn

**Affiliations:** 1 Internal Medicine, HCA Florida Bayonet Point Hospital, Hudson, USA; 2 Medicine, Edward Via College of Osteopathic Medicine, Blacksburg, USA; 3 Radiology, Medical Center of Trinity, Trinity, USA; 4 Neurology, HCA Florida Bayonet Point Hospital, Hudson, USA

**Keywords:** hemorrhagic conversion, ischemic stroke, stroke, lyme, lyme neuroborreliosis

## Abstract

Lyme disease is an infectious tick-borne illness predominant in northeastern and midwestern United States. The clinical presentation varies significantly and only a few cases develop Lyme neuroborreliosis (LNB), which makes diagnosis difficult. A 59-year-old male visiting from Michigan presented to a hospital in Florida with an ischemic stroke with aphasia and acute confusion for two days. He had imaging that noted a subacute infarct in the left parietal lobe along with multiple areas of white matter signal abnormalities and CSF serology positive for *Borrelia burgdorferi* IgM and IgG antibodies. The patient was placed on ceftriaxone for 30 days and showed significant clinical improvement. We present a case of ischemic stroke with hemorrhagic conversion and an incidental finding of LNB.

## Introduction

Lyme disease is an infectious tick-borne disease caused by *Borrelia burgdorferi*, most commonly spread by the Ixodes ticks and predominantly seen in America's northeastern and midwestern regions. It is a multisystem infectious disease, which has an incidence of 40 per 100,000 people and may affect any age group. The clinical manifestations vary from flu-like symptoms to cranial nerve palsies [1].

Three stages characterize Lyme disease, i.e., localized, disseminated, and late, based on the duration of infection and clinical manifestations. The localized stage occurs until one month and may present with nonspecific flu-like symptoms and the classic erythema migrans rash. The disseminated stage occurs from one to four months and may present with cardiac and neurological symptoms. These symptoms may include palpitations, chest pain, cranial nerve palsies, encephalopathy, and meningitis. The late stage occurs several months to years after the initial onset of infection and presents with neuropsychiatric symptoms in addition to arrhythmias, atrioventricular nodal block, hemiparesis, ataxia, autonomic dysfunction, and seizures [1].

Only 10-20% of cases develop Lyme neuroborreliosis (LNB), which may present with lymphadenopathy, cranial nerve palsies, and lymphocytic meningitis [1]. However, in extremely rare scenarios, *B. burgdorferi *infection may induce CNS vasculitis resulting in ischemic or hemorrhagic stroke [2]. We present a rare case of LNB with a concurrent ischemic stroke and hemorrhagic conversion. For this case report, the discussion will be limited to LNB.

## Case presentation

A 59-year-old male with a past medical history of atrial fibrillation on apixaban, coronary artery disease, hypertension, and type 2 diabetes mellitus presented with aphasia and acute confusion for two days. The patient was transferred to our hospital for further evaluation and treatment.

Physical exam was remarkable for lethargy, altered mentation, poor attention, and expressive aphasia. He had normal facial symmetry, muscle tone, strength bilaterally, and no meningeal signs.

Initial imaging included computed tomography (CT) of the head that showed a 2.9-cm temporoparietal hypointensity with mild surrounding vasogenic edema (Figure 1). Since the differential for this lesion included metastasis, a CT of the chest/abdomen/pelvis was ordered, which showed a complex multi-septated cystic mass within the presacral space. The cystic mass demonstrated no aggressive features and was thought to be a low-grade malignancy.

**Figure 1:** Head CT showing a 2.9-cm temporoparietal hypointensity with mild surrounding vasogenic edema (red arrows).

Magnetic resonance imaging (MRI) of the brain was performed to better visualize the lesion. MRI brain showed a subacute infarct in the left parietal lobe (Figure 2) and subependymal signal abnormalities with enhancement in the right periventricular white matter, thalamus, hippocampal tail, and bilateral occipital lobes, suspicious for neoplasm (Figure 3).

**Figure 2:** Brain MRI showing a subacute infarct in the left parietal lobe (red arrows).

**Figure 3:** Brain MRI showing subependymal signal abnormalities with enhancement in the right periventricular white matter, thalamus, hippocampal tail, and bilateral occipital lobes (grey arrows) and suspicious left neoplasm (red arrows).

In addition, a CT angiography of the neck demonstrated no vascular disease. The patient originally lived in Michigan, and he was only visiting Florida prior to hospitalization. The family reported that he may have had a rash over 10 years ago and was not evaluated by a primary care physician since the rash disappeared. Lyme disease was suspected due to the patient’s history, travel from an endemic area, and MRI findings that were remarkable for multiple foci of abnormal signal intensity in the cerebral white matter. A lumbar puncture was performed with CSF cytology that was negative for atypia, malignancy, or inflammation. CSF findings were as follows: colorless appearance, 3 WBC, 100 RBCs, 77 mg/dl of glucose, 128 mg/dl of total protein, and 78 mg/dl for albumin. CSF serologies were as follows: positive for *B. burgdorferi *IgM and IgG antibodies and varicella-zoster virus (VZV) IgG, and negative for venereal disease research laboratory (VDRL), *Cryptococcus* antigen, and herpes simplex virus (HSV) I and II. Unfortunately, we did not test for all tick-associated infections due to limited resources.

Another MRI was obtained 10 days later to reassess brain lesions, which showed an evolving hemorrhage in the left posterior parietal lobe and persistent multiple foci of abnormal signal intensity in the cerebral white matter (Figure 4). MRI findings were negative for cerebral edema or midline shift.

**Figure 4:** MRI showed an evolving hemorrhage in the left posterior parietal lobe and persistent multiple foci of abnormal signal intensity in the cerebral white matter (red arrows).

The patient was started on ceftriaxone 2 g daily for 30 days per infectious disease based on clinical presentation, imaging findings, and lab findings, as the benefits outweigh the risks for the treatment of LNB.

As the hospital course progressed, the patient began to improve in his receptive aphasia and encephalopathy. On day 14, prior to discharge, a repeat CT of the brain was negative for any evolution of the hemorrhagic conversion and the patient was alert, oriented, and could respond to questions and follow commands. The patient was discharged with appropriate medications including IV antibiotics to complete the 30-day course and instructions to follow up with their primary care provider, cardiology, neurology, oncology, and infectious disease.

Per the patient’s spouse, outpatient imaging follow-up demonstrated resolution of the white matter signal abnormalities with continued improvement in the patient's symptoms. However, a degree of receptive and expressive aphasia persists. The patient is able to meet all requirements of his job and perform all activities of daily living without assistance.

## Discussion

LNB is a rare manifestation that develops in only 10-20% of infected individuals. A systematic review of published cases in 2017 regarding the association of neuroborreliosis with stroke and vasculitis noted 88 cases globally. Only five of these cases were reported in the USA. The majority of cases are in northern European countries as the prevalence of tick-borne infections is significantly higher [2,3]. This variance in prevalence may contribute to milder nervous signs and symptoms with Lyme disease in North America [4].

Here we discuss the most common clinical manifestations and speculated pathophysiology of LNB. A retrospective study between 1999 and 2014 found 68 patients with LNB and evaluated their neurological manifestations. Results showed that the most common to least common manifestations were as follows: cranial nerve palsy, painful radiculitis, encephalitis, myelitis, and meningitis [5]. As such, stroke is a rare presentation of LNB and less than 10 case reports have been well documented with similar clinical presentations [6-9]. The pathogenesis of LNB resulting in strokes is not well defined; however, the present understanding suggests inflammation [10]. A study assessing the role of inflammation in the pathogenesis of LNB performed in rhesus monkeys showed that there is a causal role of inflammation with acute LNB [11]. A small case series of three LNB patients who were evaluated via MRI and tissue samples concluded a possible association between Lyme infection and cerebral lymphocytic vasculitis as well as multifocal encephalitis [12].

Fortunately, the majority of these patients responded well to antibiotics therapy and overall mortality was 4.7% [2]. Although there is not sufficient evidence on the pharmacological treatment of LNB due to the rarity, a systematic literature review on treatment found no significant evidence for extended antibiotic treatments greater than four weeks [13].

For this particular patient, there are multiple risk factors that increase the chance of a thromboembolic event. As a comorbid condition, LNB certainly exacerbated and worsened the clinical course of recovery. This would be the sixth reported case in the US of LNB concurrent with ischemic stroke where LNB may be determined to be causal. Furthermore, the hemorrhagic conversion and clinical improvement with antibiotic treatment certainly allow for the consideration of LNB as the causal agent.

## Conclusions

LNB is a rare presentation of Lyme disease in the USA and may be difficult to diagnose. This disease presents with great variability in clinical presentation and can worsen cerebrovascular accidents (CVAs), as seen in this patient. The association of Lyme disease with stroke is rare and the scarcity of cases makes it difficult to have a standardized treatment plan. Although LNB is not a primary consideration in acute CVA, we suggest that neuroborreliosis should be considered in the differential in patients who present with stroke or acute confusional state in endemic areas of Lyme disease.
